# Establishment of a Finite Element Model of Normal Nasal Bone and Analysis of Its Biomechanical Characteristics

**DOI:** 10.1155/2023/3783051

**Published:** 2023-03-31

**Authors:** Liuqing Zhang, XinYue Wang, Yiyuan Sun, Shuqin Wang, FuLong Zhang, Zhen Zhang

**Affiliations:** ^1^Department of Otolaryngology Head and Neck Surgery, The First Affiliated Hospital of Bengbu Medical College, Bengbu, Anhui 233000, China; ^2^Department of Ophthalmology, The First Affiliated Hospital of Anhui Medical University, Hefei, Anhui 230022, China; ^3^Department of Otolaryngology Head and Neck Surgery, ShangHai Nineth Hospital, School of Medicine, Shanghai Jiaotong University, Shanghai 200001, China; ^4^Department of Imaging, The First Affiliated Hospital of Bengbu Medical College, Bengbu, Anhui 233000, China; ^5^Department of Emergency Surgery, The First Affiliated Hospital of Bengbu Medical College, Bengbu, Anhui 233000, China; ^6^Department of Pediatric, The First Affiliated Hospital of Bengbu Medical College, Bengbu, Anhui 233000, China

## Abstract

Nasal bone is a long, paired series of small bones, which is narrow at the top and broad at the bottom, that forms the base of the nasal dorsum. Together with the nasal part of the frontal bone, the frontal process of the maxilla and the middle plate of the ethmoid bone constitute the bone scaffold of the external nose. In this paper, the DICOM image data file was imported into the Mimics software for 3D reconstruction. At the same time, the Geomagic software was used for relevant image processing, and the finite element software ANSYS was used to establish a finite element model to analyze the stress characteristics of the nasomaxillary complex. *Results*. The maximum principal stress and maximum strain force at the lower segment of nasal bone and the junction of nasal bone and maxilla were relatively large. When the same external force acts on the lower segment of the nasal bone and the angle is 0° (sagittal force), the maximum principal stress and maximum strain force are the smallest. When the angle continues to increase, the maximum principal stress and maximum strain force continue to increase.

## 1. Introduction

Nasal bone is one of the important components of maxillofacial bone cartilage scaffold. Because it independently protrudes in the center of maxillofacial region and its structure is relatively thin, it is particularly prone to fracture under the action of external force [1]. Its biomechanical mechanism is very important for understanding its biological characteristics, which is also the basis for solving related clinical problems. Normal nasal bones are divided into left and right parts, which are roughly rectangular in shape [2]. The left and right parts cannot be completely symmetrical, and the connection between them is also very close. When an external force acts on the nasal bone, it is easy to cause nasal deformity, thus affecting the appearance of the maxillofacial region, and in serious cases, it will lead to nasal ventilation disorders. Accurate and rapid establishment of a three-dimensional finite element model of nasal bone is helpful to understand its biomechanical properties and analyze its stress mechanism [3]. In recent years, the finite element method has been widely used in the related research of human limbs, spine, or various soft tissues, while the establishment of the finite element model of nasal bone and the biomechanical research are few [4]. The correlation analysis of the biomechanical characteristics of nasal bone provides a basis for the clinical diagnosis and treatment of nasal bone fracture and also lays a foundation for the related biomechanical research of otolaryngology and craniomaxillofacial surgery.

This study also has certain limitations. First of all, the number of materials collected is limited. The materials of this study are from hospitalized patients in our hospital. The selection of materials is relatively random, and there is no large-scale research, which has certain limitations. Second, the results of finite element analysis of nasal bone depend on the quality of modeling to a certain extent [5, 6]. Due to the influence of soft tissue, muscle, ligament, and other structures around the nasal bone, there is certain subjectivity in a series of processes such as image segmentation and image processing in the research process. In addition, some steps can be simplified in the modeling process, which may also lead to the model established in the research not being completely consistent with the real tissue structure characteristics. The biomechanical environment that completely simulates the nasomaxillary complex cannot be achieved at present. Finally, at present, most bone modeling still endows materials with a single modulus [7], but there is no unified evaluation standard in finite element modeling, material properties, and algorithms. The same is true in this study. The finite element model calculated through experiments is different from the substantive structural stress situation [8]. Some scholars calculate the elastic modulus of different materials based on different gray values of different bones. However, the relevant empirical formulas need to be further amended and improved.

## 2. Data and Methods

### 2.1. Modeling Data Collection

100 normal adult nasal bone imaging data were randomly collected. The patient had no history of maxillofacial trauma and surgery, and no history of related maxillofacial diseases.

### 2.2. Equipment Selection and CT Scanning Three-Dimensional Reconstruction

64 slice spiral CT was used to scan the nasal bones of healthy adults, and the CT plain scan image data of patients were obtained [9]. The scanning range is from the frontal bone to the bottom of the nose and from both sides to the lateral margin of the bilateral maxilla. The scanning layer thickness is 0.625 mm. First, the extracted imaging data are saved in DICOM (digital imaging and communications in medicine) format [10, 11]. The collected nasal bone imaging data were reconstructed by using the medical 3D reconstruction software mimics (material's interactive medical image control system) 20.0, and the appropriate gray threshold was set to segment the obtained image, establish the normal nasal bone and surrounding bone imaging model, and temporarily output it as a STL format file.

### 2.3. Postprocessing

Because the obtained STL format file is relatively rough, it is imported into Geomatic studio (American Geomatic company) for smooth noise reduction and surface processing. After relevant details are repaired, a smooth surface model is constructed. After the surface model is converted into a solid model, the file is saved in IGES format (as shown in Figure 1).

### 2.4. Establishment of Mesh Solid Model of Nasomaxillary Complex

The postprocessing three-dimensional model of nasomaxillary complex is imported into the finite element analysis software ANSYS workbench'19.0 (analysis system) [12], the boundary and contour lines of the three-dimensional solid model are established, and the tiny points, lines, and surfaces that have or may have an impact on the modeling are manually processed, and the model is divided into regular modules. When delimiting, the element size is set to 1 mm, 2 mm, and 3 mm, respectively. After repeated calibration, it is found that the 1 mm grid is the most suitable for this study. After division, the divided volume mesh is synthesized. After manual calibration, the mesh model of the nasomaxillary complex with 162086 units and 202528 nodes is finally generated (as shown in Figure 1).

### 2.5. Setting of Boundary Constraints and Stress Analysis

We treat the nasomaxillary complex as a whole, remove the constraints of surrounding soft tissue, muscles, ligaments, and other structures on the nasomaxillary complex, and fix the upper end of the nasal bone and the lateral edge of the double maxilla, and the lower end is the free edge. The nasal bone is divided into upper, middle, and lower parts (Figure 2). The upper end is the part above the level of the anterior inner segment of the frontomaxillary suture, the middle part is the narrowest part, and the lower part is from the lower segment of the medial edge of the nasal bone to the outer edge of the nasal bone.  Figure 3 shows the distribution of the maximum principal stress and strain force generated by the 100 N vertical external force at the junction of the upper, middle, and lower segments of the nasal bone and the lateral nasal bone and maxilla. It is necessary to further select the lower segment of the nasal bone to simulate the stress and strain distribution of the nasal bone under the action of 100 N external force environment at different angles of 0°, 30°, 45°, 60°, 75°, and 90° (0° parallel to the sagittal plane), as shown in Figure 4. In this study, the author refers to relevant studies to define relevant parameters and selects the elastic modulus of 137000 MPa and Poisson's ratio of 0.326.

## 3. Results

In this study, the structure of nasomaxillary complex can be vividly reproduced by modeling. After simulating the vertical stress of 100 N at the junction of the upper, middle, and lower segments of the nasal bone and the lateral nasal bone and maxilla, the results show that (as shown in Table 1) the maximum principal stress at the upper and middle segments of the nasal bone is relatively less than that at the junction of the lower segment of the nasal bone and the lateral nasal bone and maxilla, and the strain force at the upper and middle segments of the nasal bone is relatively less than that at the junction of the lower segment of the nasal bone and the lateral nasal bone and maxilla. When different angular forces are applied to the lower segment of the nasal bone (the magnitude of the force is equal to 100 N), when the angle is 0°, that is, when the direction of the force is parallel to the sagittal plane, the maximum principal stress and maximum strain force are the smallest, and when the angle is 90°, that is, when the force is perpendicular to the sagittal plane, the maximum principal stress and maximum strain force are the smallest. During this period, the angle is that with the continuous increase of the angle, the maximum principal stress and the maximum strain force are also increasing (as shown in Table 2).

## 4. Discussion

With the continuous development of biomechanics, the finite element method is gradually applied to various fields, and bone stress analysis is one of the main application fields of FEM [13, 14]. In this study, the results of FEM analysis can not only explain the biomechanical mechanism of nasomaxillary complex injury [15] but also provide some theoretical guidance for nasomaxillary complex injury in future clinical diagnosis and treatment. In this study, the stress of nasal trauma was simulated and analyzed by the finite element method [16]. Combined with the research results in Figure 3 and Table 1, it can be found that under the same external force conditions, the maximum principal stress of the upper middle segment of nasal bone is relatively less than that of the lower segment of nasal bone and the junction of lateral nasal bone and maxilla, and the strain force of the upper middle segment of nasal bone is relatively less than that of the lower segment of nasal bone and the junction of lateral nasal bone and maxilla [17]. Considering that the lower segment of the nasal bone protrudes in the center of the maxillofacial region, the structure is relatively thin, so it is relatively prone to fracture under the action of external force [18, 19]. In addition, the junction of nasal bone and maxilla, that is, the nasomaxillary suture, is the bone junction, which runs through the whole length of the lateral edge of nasal bone and the medial edge of maxilla. The bone in the suture junction area is relatively weak, and it is also prone to fracture or separation under the action of external force, and the maxillary sinus cavity of adults will become more protrusive after maturity [20]. Therefore, the maximum stress, that is, the maximum strain force, measured at the lower segment of the nasal bone; that is, the side in this study is relatively large.

Combined with the research results in Figure 4 and Table 2, it can be found that under the same external force, the maximum principal stress and maximum strain force gradually increase with the increasing angle of the lower nasal bone. Considering that when the angle is 0°, that is, when an external force is applied in the sagittal direction, the vertical external force acts directly on the nose, and the force direction is parallel to the nasal septum. As an external nasal support, the nasal septum has a certain supporting effect, and the space of the upper and lower diameters of the nasal septum suddenly decreases under the action of the external force, and the nasal septum can resolve the impact of some external forces in a deflected way to a certain extent. When the angle increases continuously, according to the principle of force decomposition, the lateral force of the external nasal bracket increases continuously. When the direction is perpendicular to the nasal bone bracket, that is, the angle is 90°, the lateral force is the largest, and the squeeze nasal bone shifts sideways, and the supporting structure of the external nasal skeleton is more likely to be damaged. At this time, the maximum principal stress of the external nose, that is, the maximum strain force, is the largest; that is, it is more prone to fracture.

## 5. Conclusion

The stress of nasal bone under the same external force at different action points and angles is studied by finite element analysis, and the combination of three-dimensional reconstruction and finite element analysis provides a certain theoretical basis for the study of the stress mechanism of nasal maxillary complex and also provides a basis for the clinical diagnosis and treatment of nasal trauma, nasal bone, and surrounding structural fractures.

## Figures and Tables

**Figure 1:** Nasomaxillary complex model and mesh model.

**Figure 2:** Positioning of the upper, middle, and lower segments of nasal bone and the junction of nose and maxilla.

**Figure 3:** Stress and strain distributions of the upper, middle, and lower nasal bone and nasomaxillary junction under 100 N vertical external force.

**Figure 4:** Distribution of stress and strain at the lower end of nasal bone at different angles.

**Table 1:** Stress and strain distributions of nasal bone and its surrounding parts.

	Maximum principal stress (PA)	Maximum strain force (mm/mm)
Upper segment	2.54	0.000243
Middle part	3.69	0.000489
Lower segment	4.02	0.000985
Flank	5.84	0.000544

**Table 2:** Stress and strain distributions of nasal bone at different angles.

	Maximum principal stress (PA)	Maximum strain force (mm/mm)
0°	4.02	0.000085
30°	6.71	0.000931
45°	13.49	0.001287
60°	19.37	0.001848
75°	23.93	0.002284
90°	26.86	0.002566

## Data Availability

The data used to support the findings of this study are included in the article.
